# Analysis of Polymorphisms in the Lactotransferrin Gene Promoter and Dental Caries

**DOI:** 10.1155/2011/571726

**Published:** 2011-12-08

**Authors:** João Armando Brancher, Giovana Daniela Pecharki, Andrea Duarte Doetzer, Kamilla Gabriella dos Santos Medeiros, Carlos Alberto Cordeiro Júnior, Vanessa Santos Sotomaior, Peter Bauer, Paula Cristina Trevilatto

**Affiliations:** ^1^Center for Health and Biological Sciences, Pontifical Catholic University of Paraná (PUCPR), Imaculada Conceição Street 1155, 80215-901 Curitiba, PR, Brazil; ^2^Department of Medical Genetics, University of Tübingen, Calwerstrasse 7, Tübingen D 72076, Germany

## Abstract

Regarding host aspects, there has been strong evidence for a genetic component in the etiology of caries. The salivary protein lactotransferrin (LTF) exhibits antibacterial activity, but there is no study investigating the association of polymorphisms in the promoter region of *LTF* gene with caries. The objective of this study was firstly to search the promoter region of the human *LTF* gene for variations and, if existent, to investigate the association of the identified polymorphisms with dental caries in 12-year-old students. From 687 unrelated, 12-year-old, both sex students, 50 individuals were selected and divided into two groups of extreme phenotypes according to caries experience: 25 students without (DMFT = 0) and 25 with caries experience (DMFT ≥ 4). The selection of individuals with extreme phenotypes augments the chances to find gene variations which could be associated with such phenotypes. *LTF* gene-putative promoter region (+39 to −1143) of the selected 50 individuals was analyzed by high-resolution melting technique. Fifteen students, 8 without (DMFT = 0) and 7 with caries experience (mean DMFT = 6.28), presented deviations of the pattern curve suggestive of gene variations and were sequenced. However, no polymorphisms were identified in the putative promoter region of the *LTF* gene.

## 1. Introduction

Dental caries is a multifactorial infectious disease that may result in loss of mineral from affected teeth [1]. The prevalence of the disease has reduced significantly, including Latin America and Brazil [2]. Nevertheless, groups of children have still been showing high levels of caries activity. This phenomenon of dental caries concentration in small groups is termed *polarization* and represents one of the epidemiological disease aspects, in which a portion of the population has focused most of the needs for treatment [3, 4]. Treatment of caries is extremely costly, representing the fourth most expensive disease to treat in most of the third world countries [5]. 

Caries disease is caused by organic acids that originate from microbial fermentation of carbohydrates from the diet [6, 7]. Beside the microflora [8, 9], cavities may appear whether cariogenic microorganisms and carbohydrates are present in a susceptible individual during a certain time in the mouth [10, 11]. Other risk factors that may influence individual susceptibility to caries development are socioeconomic status [12], oral health behavior [13, 14], gender [15], and ethnicity [16]. In addition, it seems that host response, represented by teeth and saliva, contributes to caries outcome [17].

 Saliva presents various innate and acquired defense factors capable of inhibiting bacterial invasion, growth, and metabolism by different mechanisms [18–20] such as bacterial adherence and streptococci acid production [21]. So far, researches have investigated several biological determinants, which can influence the biofilm cariogenicity [6–22], such as saliva flow and composition [20–23]. A constant salivary flow efficiently eliminates microorganisms from oral cavity; thus, a reduced flow may easily take to microbial growth, followed by teeth deterioration [1–19]. Some salivary proteins have an antibacterial effect, like lysozyme, lactoperoxidase, immunoglobulins, agglutinines, mucins, and lactotransferrin [20–24]. At the molecular level, there is a functional overlapping among several salivary proteins [18–25]. 

Lactotransferrin (LTF) is a multifunctional metalloprotein [26], belonging to the transferrin family [27, 28], with a molecular weight of about 80 kDa and 670–690 amino acid residues organized in two lobes: N and C [29]. It is expressed in several cells, such as glandular epithelial tissues and human neutrophils [27–30], and presented in diverse organism fluids, such as tears, semen, sweat, colostrum, milk, nasal secretion, and saliva [30, 31]. LTF is considered a cytokine that plays a role in the protection against several infections [31, 32] such as by fungi [32], protozoa [9], and viruses [9–34]. LTF can modulate dental biofilm aggregation and development, inhibiting *Streptococcus mutans *adhesion [35, 36]. 

Regarding host aspects, there is strong evidence for a genetic component in the etiology of caries disease [23–37]. However, little is known concerning how many and which are the genes influencing caries genetic predisposition.

*LTF* gene is localized on the human chromosomal 3p21 [38, 39], organized into 17 exons, with 24.5 kb in humans [30]. Polymorphisms are gene sequence variations whose minimum allele frequency is higher than 1% in the population, and they are distributed throughout the entire genome [40]. Catalogued single nucleotide polymorphisms (SNPs) in public databases have been growing from 1.4 million in 1999 [41] to 2.1 million in 2001 [42] up to approximately 4.1 million markers [43]. Functional polymorphisms are variations, which may (i) alter amino acid sequence in the protein sometimes affecting the function of the protein and (ii) modify the levels of transcripts and protein. Polymorphisms in regulatory sequences of the gene promoter can affect the protein function indirectly by altering its expression and RNA processing [44]. *LTF* gene polymorphisms have been described [44] and associated with aggressive periodontitis [45–47], herpes simplex keratitis [48], and dental caries [49]. However, to the authors' knowledge, there is only one report investigating the association between polymorphisms in *LTF* gene and dental caries [49], and there is no study investigating the association of polymorphisms in the promoter region of *LTF* gene with caries.

The objective of this study was firstly to search the promoter region of the human lactotransferrin gene (*LTF*) for gene variations and, if existent, to investigate the association of the identified *LTF* gene polymorphisms in this region with dental caries in 12-year-old students.

## 2. Materials and Methods

### 2.1. Sample Selection

Firstly, 687 unrelated, 12-year-old, both sex students from private and public schools of Curitiba, PR, Brazil, were diagnosed according to the decayed, missing, and filled teeth index (DMFT). All examinations were conducted by two examiners. To assess the consistency of each examiner (inter- and intraexaminer reproducibility), duplicate examinations were conducted on 10% of the sample and the Kappa test was used to measure reliability and the value of 0.93 was obtained, which indicated almost perfect reproducibility of the data. Examinations were conducted in schoolrooms in accordance with the international standards established by the WHO [50]. From those 687 students, 331 individuals were without caries experience (DMFT = 0) and 346 individuals with caries experience (DMFT ≥ 1). The students were selected for study only if the parent/caregiver returned the informed consent form, according to norms of the Ethical Committee on Research of the Center for Health and Biological Sciences of the Pontifical Catholic University of Paraná (PUCPR), according to the Resolution 196/96 of the Health National Council, register no. 487. Twelve schools were randomoly chosen, one public and one private school from each health district of the city. Students were not included if smokers, using orthodontic appliances, taking chronic anti-inflammatory and antibiotics in the last three months, or with history of any disease known to compromise immune function. 

From the selected students, the study sample was composed of fifty (*n* = 50) 12-year-old, both sex students with extreme phenotype (Table 1):

Group 1 (G1): 25 students without caries experience (DMFT = 0),
Group 2 (G2): 25 students with caries experience (DMFT ≥ 4).

The idea of selecting 50 students with extreme phenotypes, 25 without caries experience (DMFT = 0) and 25 with high caries experience (DMFT ≥ 4), was to augment the chances to find gene variations which could be associated with such phenotypes (DMFT = 0 and ≥4 were considered extreme phenotypes because the mean DMFT in Curitiba, PR, Brazil, for 12-year-old students is 1.27 [51].

### 2.2. DNA Collection

The sampling of epithelial buccal cells was performed as previously described [52]. Briefly, the individuals undertook a mouthwash after 1 min, containing 5 mL 3% glucose. Following mouthwash, a sterile wood spatula was used to scrape oral mucosa. The tip of the spatula was then shaken into the retained mouthwash solution. Buccal epithelial cells were pelleted by centrifugation at 2000 g for 10 min. The supernatant was discarded and the cell pellet resuspended in 1.300 mL of extraction buffer (10 mM Tris-HCl (pH 7.8), 5 mM EDTA, 0.5% SDS). Ten *μ*L proteinase K (20 mg/mL) was added to the solution, being left overnight at 65°C. DNA was purified by adding ammonium acetate 10 M, precipitated with isopropanol and resuspended with 50 *μ*L Tris 10 mM (pH 7.6) and EDTA 1 mM [53].

### 2.3. *LTF* Gene-Promoter Region Amplification by High-Resolution Melting (HRM)

For the PCR analysis, fifty (50) students with extreme phenotype for caries (25 DTMF = 0 and 25 DTMF ≥ 4) were selected. For the analysis, 15 *μ*L final volume of reaction was prepared with 2 *μ*L (10 ng) genomic DNA, 7.5 *μ*L LightCycler 480 High Resolution Master Mix (Roche Diagnostics, Mannheim, Germany), 0.4 *μ*L (10 pmol) of each oligonucleotide primer, 1.2 *μ*L MgCl_2_ (Roche Diagnostics, Mannheim, Germany), and 3.5 *μ*L deionizated water. Five primer pairs were used to amplify a promoter sequence in the *LTF* gene containing transcription boxes (Table 2).

The polymerase chain reaction (PCR) and melting acquisition were performed in a single run on a LightCycler 480 instrument (Roche Diagnostics, Mannheim, Germany). According to the manufacturer's instructions, it was transferred 10 *μ*L PCR product to 384-well plates suitable for HRM analysis. A centrifugation was performed as specified by the manufacturer to eliminate air bubbles that might disturb fluorescence curves. 

The PCR cycling protocol consisted of an initial heating step at 95°C for 10 minutes followed by 45 cycles of denaturation at 95°C for 10 seconds, annealing starting at 68°C for 15 seconds, and extension at 72°C for 20 seconds. After amplification, the amplicons were first heated to 95°C for 1 minute, and then the HMR program went over the range from 65°C to 95°C with 25 signal acquisitions per degree. Melting curve analysis was performed on the Light scanner with Lightscanner Software and on the LightCycler 480 with the Gene Scanning module. The software program employ a 3-step analysis: (1) normalization by selecting linear regions before (100% fluorescence) and after (0% fluorescence) the melting transition, (2) temperature shifting by moving the curves along the *x*-axis, facilitating grouping, and (3) use of the Auto Group function. To analyze sample's melting-temperature profiles, the fluorescence of the samples was monitored while the temperature of the LightCycler 480 instrument thermal block cycler had steadily increased. As the temperature increased, sample fluorescence decreased. The reaction conditions are shown in Table 3.

### 2.4. PCR and DNA Sequencing of “Cases”

Samples, whose results did not follow the standard curves, needed to be checked for polymorphisms and were termed “cases.” With the intention of sequencing the cases, PCR was carried out in a final reaction volume of 45 *μ*L, containing 1.8 *μ*L of each primer (R and F), 1.8 *μ*L DNA, and 39.6 *μ*L PCR Supermix-Invitrogen. Amplification was performed with an initial denaturation at 94°C for 5 min followed by 30 cycles of 94°C for 1 min, 58°C for 1 min, and 72°C for 1 min, with a final extension for 7 min at 72°C on a Touchgene Gradient Thermocycler (Techne, Cambridge, UK). 

The PCR products were evaluated following electrophoresis through a 1.5% agarose gel (Promega, Madison, Wis, USA), stained with ethidium bromide (Sigma), and visualized using an AlphaImager (Alpha Innotech, San Leandro, Calif, USA). Each PCR product was purified using a Genomed JETquick, PCR Product Purification spin kit (Poststra*β*e 22, 32582 Löhne, Germany). The sequencing reactions were performed by MWG-Biotech forward and reverse twice, and the sequence data were analyzed using the DNASTAR suite of programs (DNASTAR, Inc., Madison, Wis, USA).

## 3. Results

Fifty (50) students with extreme phenotype, 25 without caries experience (DMFT = 0) and 25 with caries experience (DMFT ≥ 4), were analyzed by HRM technique, whose amplification patterns can be seen in Figure 1. 

Fifteen (15) students, being 8 without and 7 with caries experience (mean DMFT = 6.28), were classified as “cases,” being further sequenced (Table 4). All the five primer pairs showed good quality results in the sequencing. An example of one sequenced sample using primer pair 5 can be observed in Figure 2. 

No polymorphisms in the study promoter region of the *LTF* gene (+39/−1143 bp) were identified.

## 4. Discussion

Although dental caries has been declining recently [54], it is still a major public health concern worldwide [50]. It has an impact on individuals and communities by leading to tooth loss and dental pain, resulting in suffering, impairment of function, reduced quality of life, and absenteeism at school and work [1–50].

The etiology of dental caries has been studied for many years. Multiple factors may be contributing to a person's risk to caries, including three essential interactive factors: host such as saliva properties and tooth enamel surface, biofilm, and diet [55], with the addition of another factor: time [56]. More recently, environmental, such as socioeconomic status [57], and oral health behavior [14] and genetic aspects [58] have also been related to caries etiology.

In spite of all that has been known about this disease, there are still individuals who appear to be more susceptible to caries and those who are extremely resistant, regardless of the environmental risk factors to which they are exposed [59]. Recently, our group showed for the same study sample that the DMFT index was significantly higher (2.88) among the students with caries experience than those for the whole sample (1.46) (unpublished data). This finding evidenced the polarization phenomenon in the study sample and points to an individual host response modulation influencing caries outcome. 

Based on the multifactorial nature of dental caries, it has been suggested that susceptibility or resistance to caries would be the result of one or more gene-environment interactions [59]. Studies have identified a strong genetic component controlling susceptibility to caries [60]. Hereditary aspects of caries have been discussed since the 1920s [61]. Firstly, the studies investigated genetic aspects related to cariogenic bacteria [62]. Nowadays, genetic analyses report aspects associated with individual susceptibility to dental decay development [37–63]. There have been pieces of evidence associating hereditary aspects with dental caries, such as familial aggregation studies [64]. Gold standard studies aiming to dissect the genetic component underlying a given complex disease such as caries are (i) twin studies [65–67] and (ii) complex segregation analysis (CSA) [68]. Twin studies, which compare concordance rates between monozygous and dyzigous twins, have shown that between 50 and 70% of the phenotype variation are explained by genes [66, 67], while the CSA detected a dominant major gene effect which best explained the phenotype. However, these kinds of analyses fail to identify how many and which genes underlying the controlling of susceptibility to diseases are [68].

 Candidate genes underlying host susceptibility to caries could range from (1) genes contributing to enamel formation [69], (2) to those for saliva composition [49], and (3) immune response [70]. Concerning saliva, several studies have been investigating salivary proteins involved in modulating biofilm aggregation and adhesion, buffer capacity, and other qualitative aspects of saliva [19–72]. 

The salivary protein LTF exhibits bactericidal and bacteriostatic activity against a wide range of gram-negative and gram-positive bacteria due to its ability to chelate iron, which is essential for microbial growth and metabolism [73]. Specifically, LTF may interfere with *Streptococcus mutans* aggregation, adhesion, and biofilm development [39–74]. In addition, LTF exhibits non-iron-dependent antibacterial properties [9–36] and antifungal, antiviral, antitumor, anti-inflammatory, and immunoregulatory activities [75–78]. 

Results involving *LTF* gene and dental caries are scarce. To the authors' knowledge, there is only one report investigating the association between polymorphisms in *LTF* gene and dental caries [49]. This study found an association of a polymorphism in the second exon of *LTF* gene with lower values of DMFT, as well as with higher levels of salivary flow. The same polymorphism failed to associate with localized aggressive periodontitis, but did associate with antibacterial activity against *S. mutans*, a main cariogenic bacterium [45].

To understand the molecular mechanisms of *LTF* gene expression and regulation, it is necessary to characterize its genetic regulatory regions in the promoter. The human *LTF* putative gene promoter presents nearly 1000 bp, and several transcription factors binding sites have been involved in the positive or negative regulation of *LTF* gene expression and transcriptional activity (Figure 3). 

The purpose of this study was to characterize the putative promoter region of *LTF* gene aiming to identify variations which could affect LTF expression and biological functions, such as iron-binding and bacteria-killing abilities, which could be associated with dental caries.

In this work, five oligonucleotide primer pairs were made to amplify all the putative promoter region (+39 to −1143), which presents an abundance of identified transcription factor binding sites, in subjects with and without caries experience, intending to further associate variations in this region with caries susceptibility. Fifty samples were then analyzed by high-resolution melt (HRM) (LightCycler 480), which was able to detect different melting profiles in the sample. HRM appears to be a sensitive, robust mutation-scanning technique that could significantly reduce the time and cost of screening for mutations/polymorphisms [79]. For the 50 students analyzed, 15 individual curves from 8 without and 7 with caries experience subjects were identified as outstanding by HRM, and the sequences needed to be sequenced by MWG-Biotech. The sequencing analysis revealed that no polymorphisms in the promoter region of *LTF* gene (+39/−1143 bp) were identified.

We examined the GenBank database (NCBI, 2010) for polymorphisms within the study promoter, region and five gene sequence variations were found (rs67994108 (position −41), rs28365893 (position −232), rs4637321 (position −420), rs35869674 (position −489), rs5848800 (position −696)). However, none of them is validated by frequency. These findings are reinforced by the Teng and Gladwell [44] study, which reported a total of 7 SNPs in the human *LTF* gene promoter: at −261, −374, −401, −421, −1010, −1119, and −1261 positions, being only polymorphism −1010 (ATAT/-) frequent. In that study, 91 healthy donors of different ethnicities were used to search for polymorphisms in the exons and promoter region of *LTF *gene. In the position −261, the C to T change might affect the methylation status at the CpG dinucleotides. Furthermore, the SNPs at −374, − 401, and −421 are clustered around hormone response elements and the GATA element and might affect transcription-factor interaction at these sites, influencing the expression levels of the LTF. 

*LTF* gene is highly conserved among different species [31]. The number of amino acids encoded by 15 of the 17 exons in these species is identical, and,in 12 intron-exon splice junctions, they have identical codon interruptions. Comparing the *LTF* gene promoters from different species, common characteristics are observed. The human, mouse, bovine, porcine, and bubaline promoters are very similar in terms of number and position of transcription boxes, especially between humans and mice [31]. The fact of being extremely conserved among species and widely expressed in diverse human body tissues [80] and body fluids [81] highlights LTF as an important functional protein involved in several aspects of body homeostasis. These aspects related to LTF properties may partially explain the failure in identifying gene variations in the hotspot regions of the *LTF* regulation, in spite of the significant sample size and genetic admixture of the Brazilian population, which could impact significantly biological functions. In this context, the regulation might be controlled more by different transcriptional factors (depending on the tissue) than by gene variations.

Common diseases are usually interpreted to be caused by the additive effects of several common gene variances. However, rare variations also could be playing a role in modulating the susceptibility of those complex diseases. Thus, if this is the case for caries, 100 chromosomes, which is considered in general a good opportunity to identify common variations (termed polymorphisms), may not be sufficient and sample should be significantly augmented. 

Dental caries is a complex, multifactorial disease, and many gene variations and gene-environment interactions may contribute to its outcome [59]. Thus, as LTF is considered a pleiotropic protein involved in different aspects of caries etiopathology, the investigation of polymorphisms capturing the information of the gene as a whole may be desirable. In this context, future studies should include the analyses of tag SNPs, which are a small number of polymorphisms in linkage disequilibrium (LD), which capture the information of other polymorphisms present in the same *bins* (refined LD blocks).

In summary, no polymorphisms were identified in the putative promoter region (+39 to −1143) of *LTF* gene. As LTF is an important multifunctional protein, studies should be conducted, analyzing *bins* which may capture the whole gene information, to better understand the contribution of this gene in caries etiopathogenesis.

## Figures and Tables

**Figure 1:** Comparative sequence analysis of the promoter region amplified by polymerase chain reaction (PCR) whose melting outcome was performed in a single run on a LightCycler 480 instrument (Roche Diagnostics, Mannheim, Germany). Fifteen (15) individuals, being 8 without and 7 with caries experience (mean DMFT = 6.28), were classified as “cases,” being further sequenced.

**Figure 2:** Comparative sequence analysis of the promoter region amplified by primer pair 5. (a) Consensus sequence of the *LTF* gene, (b) individual 6 (DMFT = 0), and (c) individual 11 (DMFT = 6). There was not difference between the individual sequences of the promoter region.

**Figure 3:** Promoter region (+39 to −1143 bp) of the human *LTF* gene and transcription boxes: (a) **M** **y** **b** ^1^, **S** **P**1^2^, **C**/**E** **B** **P** ^3^, **E** **T** **s** ^4^, and **S** **P**1^5^ (region –35 to –85) are involved in LTF expression during myeloid differentiation [82]. (b) **E** **R** **E** ^6^, **C** **O** **U** **P** ^7^, and **G** **A** **T** **A**-1^8^ (region –340 to –372), a highly conserved estrogen response element (ERE) overlapping with a chicken ovalbumin upstream promoter (COUP) element [83]. (c) **S** **F** **R** **E** ^9^  and **C** **O** **U** **P** ^10^ (region – 377 to –394), an extended estrogen response element half site in addition to the *ERE*, which renders the human *LTF* gene extremely responsive to estrogen stimulation [83]. (d) **T** **A** **A** **C** **C** ^11^, a highly conserved silencing factor (–774 to –778) that binds the CCAAT displacement protein (CDP/cut) [84].

**Table 1:** Baseline characteristics of the study population.

Variables	G1 (*n* = 25)	G2 (*n* = 25)	*P* value*
	*n* (%)	*n* (%)	
Ethnic group			
Caucasian (46)	25 (100.0)	21 (84.0)	0.145
Afro-American (3)	0 (0)	3 (12.0)	
Asian (1)	0 (0)	1 (4.0)	

Gender			
Female (28)	16 (64.0)	12 (48.0)	0.254
Male (22)	9 (36.0)	13 (52.0)	

*Chi-square, *P* < 0.05.

**Table 2:** Sequence of oligonucleotide primers used for DNA amplification and the amplified promoter regions with their transcription sites.

Primer	Primers' sequences	Region	Transcription boxes
1	Sense 5-GAGGAACAGCAGGACGAG-3	+70/−188	*TATA, Myb, SP1, C/EBP, Ets, SP1 *
	Antisense 5-AGAGGAAAGCCAGCCTGC-3		
2	Sense 5-AGGCAGGACAGGACTCCAC-3	−142/−412	*ERE, COUP, GATA-1*
	Antisense 5-AAGGTGCCTAGGAGCCAGTT-3		
3	Sense 5-ATCGCCTTGACCTGTGAGAC-3	−346/−653	*SFRE, COUP*
	Antisense 5-CAAGGCTGGTTCCATGTTCT-3		
4	Sense 5-AGGGACCTCAGAGGGGAAT-3	−605/−878	*TAACC*
	Antisense 5-CGTAAATACATTCCCATGACACA-3		
5	Sense 5-AACAATCGCCATAAATGTCAG-3	−810/−1100	*TAACC*
	Antisense 5-TGGATGTGAACTTAGCCCAAGAG-3		

**Table 3:** Reaction conditions for melting acquisition performed by LightScanner and LightCycler 480.

Program/cycles	Temperature
Preincubation/01	Initial heating: 95°C
Amplification/45	Denaturation: 95°C
	Annealing: 68°C
	Final Extension: 72°C
High-resolution melting/1	Heating: 95°C
	Hybridzation: 40°C
	Melting acquisition: 65°C to 95°C
Cooling/1	40°C

**Table 4:** Baseline characteristics of the fifteen (15) students classified as “cases” being further sequenced, being 8 without and 7 with caries experience (mean DMFT = 6.28).

Variables	G1 (*n* = 8) DMFT = 0	G2 (*n* = 7) DMFT = 6.28 ± 1.7)
	*n* (%)	*n* (%)
Ethnic group		
Caucasian	8 (100)	7 (100)

Gender		
Female	7 (87.5)	4 (57.14)
Male	1 (12.5)	3 (42.86)
